The article "Correlation Analysis of Inflammatory Markers CRP and IL-6 and Postoperative Delirium (POD) in Elderly Patients: A Meta-Analysis of Observational Studies" was retracted in 2023. Reasons: suspected computer-generated content; unreliable results or conclusions; concerns about the data; concerns about the results or conclusions.

# Correlation Analysis of Inflammatory Markers CRP and IL-6 and Postoperative Delirium (POD) in Elderly Patients: A Meta-Analysis of Observational Studies

**DOI:** 10.1155/2022/1136386

**Published:** 2022-11-19

**Authors:** Xiaoling Huang, Lanyang Li, Qiuping Feng

**Affiliations:** ^1^Department of Anesthesiology, First People's Hospital of Longquanyi District, West China Hospital Sichuan University, Chengdu, Sichuan 610100, China; ^2^Department of Anesthesiology, Traditional Chinese Medicine Hospital of Longquanyi, Longquanyi Hospital of Chengdu University of Traditional Chinese Medicine, Chengdu Sichuan 610100, China

## Abstract

**Background:**

Postoperative delirium (POD) is very common in the elderly surgical population, and its occurrence is associated with multiple factors such as preoperative, intraoperative, and postoperative factors, and the increase of serum inflammatory markers such as C-reactive protein (CRP) and interleukin-6 (IL-6) is considered to be associated with the occurrence of POD, but the results of multiple studies are inconsistent. In this study, we investigated the correlation between inflammatory markers CRP and IL-6 and POD in elderly patients by literature search and meta-analysis.

**Methods:**

We searched PubMed, Web of Science, the Cochrane library, Embase, Ovid, and Springer Link for cohort studies or case-control studies that investigated the factors involved in the occurrence of POD, used the Newcastle-Ottawa Scale (NOS) to assess the quality of the selected literature, and combined the differences in serum CRP and IL-6 levels between POD and non-POD patients after surgery to evaluate the predictive value of CRP and IL-6 for the occurrence of POD.

**Results:**

This research comprised 16 papers for quantitative analysis, with a total of 2967 patients, 758 with POD and 2209 with non-POD. There were 16 cohort studies (100%) and 0 case-control studies (0%) across all the collected literatures; there were 15 prospective cohort studies and 1 retrospective cohort research. A meta-analysis revealed a statistically significant difference in serum IL-6 levels between POD patients after surgery and non-POD patients [MD = 115.68, 95% CI (25.70, 206.66), *Z* = 2.52, *P* = 0.012], as well as a statistically significant difference in serum CRP levels [MD = 27.67, 95% CI (12.77, 42.58), *Z* = 3.64, *P* = 0.0003]. *Discussion*. Early after surgery, serum IL-6 and CRP levels were considerably higher in POD patients than in non-POD patients, indicating that early serum inflammatory variables are likely to be predictors of POD. After surgery, the levels of the aforementioned inflammatory factors should be actively monitored to forecast the emergence of delirium, and active treatment should be used to limit the creation and release of the aforementioned inflammatory factors.

The article "Correlation Analysis of Inflammatory Markers CRP and IL-6 and Postoperative Delirium (POD) in Elderly Patients: A Meta-Analysis of Observational Studies" was retracted in 2023. Reasons: suspected computer-generated content; unreliable results or conclusions; concerns about the data; concerns about the results or conclusions.

## 1. Introduction

Postoperative delirium (POD) occurs within about 1 to 7 days in the early postoperative period and is a common cerebral comprehensive complication after surgery, manifested as low level of consciousness, distraction, drowsiness, apathy, and slowness of movement, and some patients experience aggressive behavior [1–3]. Study has shown that in the elderly population over 60 years of age, the proportion of POD after major surgery is about 20% to 40% [4]. However, there is no consistent understanding of the pathogenesis of POD in the elderly population, and it is only understood that POD is the result of a combination of factors, which can be divided into three parts according to the chronological order of its appearance during the pathogenesis: preoperative factors, intraoperative factors, and postoperative factors [5, 6]. Preoperative factors are related to the patient's own condition and are not easily affected by peripheral factors; intraoperative factors are related to intraoperative surgical factors and anesthesia management, which can be reduced or avoided by certain intervention measures; and postoperative factors are related to the management of postoperative rehabilitation stage of patients—pain is an important risk factor for delirium, the more severe the pain, the greater the trauma to the body, the higher the risk of delirium [7]. Abnormal stress response after surgery in patients leads to transfer of proinflammatory factors from the innate immune system and significantly increased leukocyte levels, which are thought to be directly related to the development of POD [8]. However, the results of such studies are currently controversial. In a study by Xiang et al., the researchers retrospectively compared serum IL-6 levels 1 day after surgery between POD patients and non-POD patients and found no significant difference (48.7 ± 14.8 vs 44.9 ± 16.2, *P* = 0.196) [9]. However, in another study by Chen et al., 85 elderly patients who developed POD after coronary artery bypass graft surgery were significantly different from 181 patients with non-POD in serum IL-6 levels at 6 h, 12 h, and 18 h after surgery, and the influence of postoperative IL-6 on the occurrence of POD after regression analysis was OR = 5.83, 95% CI (1.85, 18.4) [10]. The results of these studies are significantly different, and the results of multiple studies can be combined to obtain more reliable evidence by meta-analysis. Therefore, we performed this meta-analysis.

## 2. Materials and Methods

### 2.1. Database and Search Strategy

We searched the databases PubMed, Web of Science, the Cochrane library, Embase, Ovid, and Springer Link for POD-related articles, and we included all articles from all inception to March 2022 and performed electronic searches with a keyword combination “IL-6/interleukin 6” and/or “CRP/C-reactive protein” and/or “POD/Post-operative delirium”.

The article "Correlation Analysis of Inflammatory Markers CRP and IL-6 and Postoperative Delirium (POD) in Elderly Patients: A Meta-Analysis of Observational Studies" was retracted in 2023. Reasons: suspected computer-generated content; unreliable results or conclusions; concerns about the data; concerns about the results or conclusions.

### 2.2. Literature Screening Criteria

#### 2.2.1. Inclusion Criteria

(i) *Study Type*. All literatures were observational studies, including cohort study and case control study. We did not limit whether the literatures were prospective or retrospective studies

(ii) *Study Subjects*. The study subjects were elderly surgical patients. The age range and average age of the included study participants must be described in the literature

(iii) *Intervention Type*. All patients underwent some kind of surgical intervention, and we did not limit the type of surgery to tumor surgery, cardiovascular surgery, lumbar surgery, and hematologic surgery. Serum samples were collected from participants early after surgery (0 to 3 days) to determine serum IL-6 and CRP *P* values; POD was diagnosed within 7 days after surgery [11]. In the literature, participants must be divided into POD patients and non-POD patients, and the indicators must be compared

#### 2.2.2. Exclusion Criteria

(i) Exclude individual case studies, multicase studies, RCTs, reviews, and meeting minutes

(ii) Exclude the study subjects from infants, adolescents, and adults

(iii) Exclude the literature only containing cerebrospinal fluid IL-6 or CRP but no serum IL-6 and CRP

(iv) Studies lacking outcome indicators or with no data were excluded

### 2.3. Literature Screening

After retrieval and manual removal of literatures, the literatures were imported into the software NoteExpress for unified management, and repeated literatures were excluded using the deduplication function of the software. Two researchers read the titles and abstracts for further deduplication. If the titles and research contents were significantly repeated, literatures with better quality and more complete data were retained. The selected articles were further screened according to the established inclusion and exclusion criteria. If the original text cannot be obtained from the Internet, contact the author of the original text by telephone or email; if the original text cannot be obtained, the literature will be excluded. After being completed independently, the two researchers conducted cross-examination and discussion. If the inclusion of literatures was controversial, it was handed over to the third person for arbitration.

### 2.4. Literature Quality Evaluation and Risk of Bias Assessment

Newcastle-Ottawa Scale (NOS) was used to analyze the quality of the included literatures [12]. The scale was used to evaluate the object selection, comparability, and outcome indicators of the literatures. The maximum score was 9 points, and the score of more than 5 points was considered as good quality. A higher score indicates better literature quality and less bias.

The article "Correlation Analysis of Inflammatory Markers CRP and IL-6 and Postoperative Delirium (POD) in Elderly Patients: A Meta-Analysis of Observational Studies" was retracted in 2023. Reasons: suspected computer-generated content; unreliable results or conclusions; concerns about the data; concerns about the results or conclusions.

### 2.5. Data Extraction and Analysis

Two researchers independently extracted literature data: study type, location, patient age, height, weight, BMI, gender ratio, surgical methods, intraoperative indicators, cohort groups, number of cases in each group, and serological indicators. After data extraction was completed by both researchers, each other's results were cross-checked and discrepancies were discussed and finalized.

### 2.6. Outcome Indicators and Data Transformation

In this study, only IL-6 and CRP serum measurements in the early postoperative period were included, and preoperative parameters were not counted. IL-6 was measured in pg/mL and CRP was measured in mg/L. If units reported in the literature differ from statistical units, they are converted to statistical units; if CRP is reported in the literature as mg/dL, it is converted to mg/L ×10.

### 2.7. Statistical Methods

(i) Effect sizes were reported using mean variance (SMD) and 95% CI for continuous variables, using a random-effects model, and significance was judged by *Z* test and two-sided *P* value, with *P* < 0.05 indicating statistical significance; (ii) literature heterogeneity was checked by *Q* test, and *P* < 0.05 indicates heterogeneity between literatures; (iii) if heterogeneity analysis suggests heterogeneity between literatures, subgroup analysis was used to investigate the source of heterogeneity; (iv) influence analysis was performed and outlier was filtered out, and the effect size was recounted after removal [13]; (*v*) funnel plot was used to represent publication bias, and Egger's test was used to test whether the funnel plot was symmetrical

## 3. Results

### 3.1. Literature Screening Process and Results

The flow chart of literature selection (based on the process recommended by PRISMA) is shown in Figure 1, and finally 16 articles were included in the quantitative analysis.

### 3.2. Basic Characteristics of Literatures

16 articles were included in this study, including 16 cohort studies (100%) and 0 case control study (0%). There were 15 prospective cohort studies and 1 retrospective cohort study, as shown in Table 1.

### 3.3. Literature Quality and Bias Evaluation

In this study, the cases included in the literatures [9, 10, 14–27] were representative, the potential risk of bias was small, and some literatures did not describe the dropout cases in detail [22, 23], but the overall quality score of all literatures was 7-9 points, with good quality, as shown in Table 2.

The article "Correlation Analysis of Inflammatory Markers CRP and IL-6 and Postoperative Delirium (POD) in Elderly Patients: A Meta-Analysis of Observational Studies" was retracted in 2023. Reasons: suspected computer-generated content; unreliable results or conclusions; concerns about the data; concerns about the results or conclusions.

### 3.4. Meta-Analysis Results

#### 3.4.1. Comparison of Serum IL-6 Levels (pg/mL) in Patients with POD and Non-POD after Surgery

Seven literatures [10, 14–16, 18–20] reported the serum IL-6 level of POD patients and non-POD patients in the early stage after operation, unit in pg/mL, and analyzed the heterogeneity between literatures (*χ*^2^ = 416.33, *P* < 0.01). Using the random-effects model and meta-analysis showed that the difference of serum IL-6 level between POD patients and non-POD patients after operation was statistically significant [MD = 115.68, 95% CI (25.70, 206.66), *Z* = 2.52, *P* = 0.012], as shown in Figure 2.

#### 3.4.2. Comparison of Serum CRP Levels (mg/L) in Patients with POD and Non-POD after Surgery

11 literatures [9, 15, 17, 19, 21–27] reported the serum CRP level of POD patients and non-POD patients in the early stage after operation and analyzed the heterogeneity between the literatures in mg/L (*χ*^2^ = 191.74, *P* < 0.01). Using the random-effects model and meta-analysis showed that there was a significant difference in serum CRP level between POD patients and non-POD patients after operation [MD = 27.67, 95% CI (12.77, 42.58), *Z* = 3.64, *P* = 0.0003], as shown in Figure 3.

#### 3.4.3. Analysis of Source of Heterogeneity

In the analysis of serum CRP level, 11 included literatures have statistical heterogeneity (*P* < 0.01) and were divided into “tumor surgery” subgroup and “nontumor surgery” subgroup according to the type of surgery; the former included 4 literatures and the latter included 7 literatures, resulting in *P* = 0.28 for heterogeneity between groups, while heterogeneity within the two subgroups remained significant, as shown in Figure 4.

#### 3.4.4. Regression Analysis

In the analysis of serum IL-6 levels, “sample size,” “age,” and “serum collection time” were applied as independent variables, and regression analysis of the combined effect size results revealed that the regression test value obtained by sample size was *P* < 0.0001, which was statistically significant, as shown in Figure 5.

#### 3.4.5. Influence Analysis

In the analysis of serum CRP level, the influential diagnostic analysis was performed, and it was found that the literature [15] had the greatest influence on the results, and the significance of the results was not changed after removing the literature [15], indicating that this meta-analysis had good stability, as shown in Figure 6.

#### 3.4.6. Publication Bias Analysis

In the analysis of serum CRP levels, funnel plots showed uneven distribution on both sides of the funnel, suggesting publication bias, Egger's test *P* = 0.017, confirming asymmetry on both sides of the funnel, as shown in Figure 7.

The article "Correlation Analysis of Inflammatory Markers CRP and IL-6 and Postoperative Delirium (POD) in Elderly Patients: A Meta-Analysis of Observational Studies" was retracted in 2023. Reasons: suspected computer-generated content; unreliable results or conclusions; concerns about the data; concerns about the results or conclusions.

## 4. Discussion

POD can manifest as impairment of working memory, long-term memory, information processing, attention, or cognitive ability, adversely affecting quality of life, social independence, and increasing the risk of death in patients, while annual surgical patients have a higher risk of morbidity [28]. Therefore, it is very important to identify the pathogenesis and influencing factors of POD in elderly patients for the early identification of POD and to prevent the occurrence of POD after surgery in elderly patients [29]. Current research hotspots suggest that POD is associated with increased expression of proinflammatory cytokines such as CRP, IL-6, and TNF-*α*. Therefore, we performed this meta-analysis.

In this meta-analysis, we identified 16 relevant articles by electronic search, with a total of 2967 participants, 758 patients developed POD, and 2209 patients with non-POD after surgery. The combined results of 7 articles showed that the serum IL-6 level in POD patients after surgery was significantly higher than that in non-POD patients; the combined results of 11 articles showed that the serum CRP level in POD patients after surgery was higher than that in non-POD patients. This reflects that in the early postoperative period, the level of inflammatory factors in POD patients is significantly higher than that in non-POD patients, because the diagnosis of POD occurs 1 day to 7 days after surgery, and early serum inflammatory factors (within 1 day after surgery) are likely to be predictors of POD. Because the occurrence of delirium is associated with many known factors, such as preoperative psycho-psychological factors, advanced age, preoperative cognitive dysfunction, and the use of anesthetics [30], the presence of inflammatory factors may increase the chance of POD. The mechanism by which changes in inflammatory factors are associated with the development of postoperative delirium may lie in surgery is an invasive procedure, which can cause greater irritation to the patient's body, which in turn activates the immune system, leading to a strong peripheral inflammatory response and increasing the levels of multiple inflammatory factors; such cytokines can act directly or indirectly on the central nervous system, causing a secondary inflammatory response, which leads to altered cognitive function, leading to the emergence of delirium [31]. Inflammatory factors can directly interfere with neural activity and synaptic junction function in patients, such as high levels of IL-1*β* in the hippocampus can reduce synaptic plasticity, hinder potential transmission, and lead to impaired learning and memory function in patients; elevated TNF-*α* levels can also stimulate nerve cells other than neurons in the brain, regenerate actin, present degenerative changes in the nervous system, and induce the production of POD [32]. Therefore, active monitoring of the levels of the above inflammatory factors after surgery plays a role in predicting delirium, considering that nonsteroidal anti-inflammatory drugs can inhibit the formation and release of the above inflammatory factors, and timely application of drug intervention after surgery can prevent the occurrence of POD to a certain extent [33].

The article "Correlation Analysis of Inflammatory Markers CRP and IL-6 and Postoperative Delirium (POD) in Elderly Patients: A Meta-Analysis of Observational Studies" was retracted in 2023. Reasons: suspected computer-generated content; unreliable results or conclusions; concerns about the data; concerns about the results or conclusions.

In this study, when the results of multiple literatures were combined for meta-analysis, it was found that there was significant heterogeneity among literatures. We investigated the source of heterogeneity and performed subgroup analysis for literatures. However, the source of heterogeneity could not be determined. Literature heterogeneity may be related to various factors such as basic characteristics of patients included in different studies—type of surgery. Therefore, when performing pooling, we introduced a random-effects model to contain heterogeneity between different literatures.

We also performed regression analysis for factors that may affect the results and found that the sample size may directly affect the effect size MD that means the larger the sample size, the larger the resulting MD; that means the larger the difference in serum IL-6 between POD patients and non-POD patients. Because of possible errors caused by small sample sizes, we believe that studies with large sample sizes have more credible results.

In the analysis of publication bias, we noticed significant asymmetry between the left and right sides of the funnel plot (confirmed by Egger's test), which suggests that there may be publication bias in this study, because only postoperative IL-6 and CRP were included in the study, excluding the literatures reporting preoperative and intraoperative inflammatory factor levels. In addition, some literatures failing to obtain the full text and useful data were also excluded, and those with too low literature quality were also excluded, which may cause some literatures reporting negative MD to be excluded, thus causing publication bias. However, the results of many studies also showed that the increase of IL-6 and CRP before surgery was also a risk factor for POD after surgery [34–36].

Nevertheless, the 16 observational studies included in this study had a total score of more than 7 points as assessed by the NOS methodology and were good quality, and the influence analysis showed that the results were stable, suggesting that the results of this study were credible. However, studies on this topic still need to be further explored with larger sample sizes.

The article "Correlation Analysis of Inflammatory Markers CRP and IL-6 and Postoperative Delirium (POD) in Elderly Patients: A Meta-Analysis of Observational Studies" was retracted in 2023. Reasons: suspected computer-generated content; unreliable results or conclusions; concerns about the data; concerns about the results or conclusions.

A total of 2967 patients in 16 literatures were included in this meta-analysis. The results showed that the serum IL-6 and CRP levels in POD patients were significantly higher than those in non-POD patients in the early postoperative period, suggesting that the early serum inflammatory factors are likely to be predictors of POD. The levels of the above inflammatory factors should be actively monitored after surgery to predict the occurrence of delirium, and active medication should be used to inhibit the formation and release of the above inflammatory factors. Although the results of this study were stable, preoperative inflammatory factors were not considered, and the sample size was small and remains to be studied in depth. Also postoperative psychotic symptoms could be related to many other factors like perioperative pain, which deserves further exploration too [37].

## Figures and Tables

**Figure 1:** Literature selection flow chart.

**Figure 2:** Comparison of serum IL-6 levels (pg/ml) between POD patients and non-POD patients after surgery.

**Figure 3:** Comparison of serum CRP levels (mg/l) between POD patients and non-POD patients after surgery.

**Figure 4:** IL-6 subgroup analysis.

**Figure 5:** IL-6 regression analysis: sample size, age, and serum collection time.

**Figure 6:** Influence analytic.

**Figure 7:** Funnel plot analysis.

**Table 1:** Basic characteristics, grouping characteristics, and influencing indicators of included literatures.

Author and publication date	Study design	Patients number	Mean age (year)	Surgery type	Case/control PODs	Inflammatory markers	Blood sample collect point (after operation)
Xiang et al. [9]	Prospective cohort study	160	70.1	Laparoscopic surgery for colon carcinoma	39/121	CRP	Day 1
Chen et al. [10]	Prospective cohort study	266	62 ± 8.3	Coronary artery bypass graft	85/181	IL-6	18 h
Li et al. [14]	Prospective cohort study	37	60	Total hip-replacement surgery	17/20	IL-6, S-100b, TNF-*α*	1 h
Brattinga et al. [15]	Prospective cohort study	311	72 (range 65-89)	Oncologic surgery	38/273	CRP, IL-1*β*, IL-6, IL10	1 h
Lv et al. [16]	Prospective cohort study	221	52.81 ± 10.75	Acute type A aortic dissection patients treated with open surgical repair	31/190	IL-6	24 h
Cereghetti et al. [17]	Prospective cohort study	618	67 (range 59-74)	Cardiac surgery	244/374	CRP	24 h
Plaschke et al. [18]	Prospective cohort study	114	73.3 ± 6.0	Open-heart cardiac surgery	34/80	IL-6	1 h
Neerland et al. [19]	Prospective cohort study	60	84	Hip fracture surgery	46/14	CRP, IL-6	24 h
van Munster et al. [20]	Prospective cohort study	98	84.6 ± 7.1	Hip fracture surgery	50/48	IL-6	24 h
Plas et al. [21]	Prospective cohort study	136	60 (range 50-76)	Cytoreductive surgery	38/98	CRP	24 h
Khan et al. [22]	Prospective cohort study	71	62.6 (range 52.9-69.3)	Esophagectomy	26/45	CRP	24 h
Ren et al. [23]	Prospective cohort study	206	57.7 ± 11.3	Cervical or lumbar surgery	12/194	CRP	Within 2 days
Pol et al. [24]	Prospective cohort study	277	69 ± 11	Vascular surgery	16/261	CRP	Within 5 days
Slor et al. [25]	Prospective cohort study	121	85.4 ± 5.6	Hip fracture surgery	41/80	CRP	Day1~day5
Hasegawa et al. [26]	Retrospective cohort study	188	67.4 ± 12.9	Oral cancer surgery	29/159	CRP	Day 3
Pan et al. [27]	Prospective cohort study	83	71.4 ± 4.6	Lumbar spine surgery	12/71	CRP	24 h

Abbreviations: POD: postoperative delirium; IL-6: interleukin-6; CRP: C-reactive protein; TNF-*α*: tumor necrosis factor-*α*.

The article "Correlation Analysis of Inflammatory Markers CRP and IL-6 and Postoperative Delirium (POD) in Elderly Patients: A Meta-Analysis of Observational Studies" was retracted in 2023. Reasons: suspected computer-generated content; unreliable results or conclusions; concerns about the data; concerns about the results or conclusions.

**Table 2:** Quality assessment based on Newcastle-Ottawa Scale (NOS).

Literature	Case selection (/4)	Comparability (/2)	Outcome indicators (/3)	Total (/9)
Xiang et al. [9]	4	2	3	9
Chen et al. [10]	4	2	2	8
Li et al. [14]	4	2	2	8
Brattinga et al. [15]	4	2	3	9
Lv et al. [16]	4	1	2	7
Cereghetti et al. [17]	4	1	2	7
Plaschke et al. [18]	4	1	2	7
Neerland et al. [19]	4	2	2	8
van Munster et al. [20]	4	2	3	9
Plas et al. [21]	4	2	2	8
Khan et al. [22]	4	1	2	7
Ren et al. [23]	3	2	1	6
Pol et al. [24]	3	2	2	7
Slor et al. [25]	3	2	3	7
Hasegawa et al. [26]	4	2	2	8
Pan et al. [27]	4	2	3	9
